# Improvement of Sensitivity of Pooling Strategies for COVID-19

**DOI:** 10.1155/2021/6636396

**Published:** 2021-10-13

**Authors:** Hong-Bin Chen, Jun-Yi Guo, Yu-Chen Shu, Yu-Hsun Lee, Fei-Huang Chang

**Affiliations:** ^1^Department of Applied Mathematics, National Chung Hsing University, Taichung 40249, Taiwan; ^2^Department of Mathematics, National Taiwan Normal University, Taipei 11677, Taiwan; ^3^Department of Mathematics, National Cheng Kung University, Tainan City 701, Taiwan; ^4^Graduate School of Informatics, Kyoto University, Japan; ^5^Division of Preparatory Programs for Overseas Chinese Students, National Taiwan Normal University, New Taipei City 24449, Taiwan

## Abstract

Group testing (or pool testing), for example, Dorfman's method or grid method, has been validated for COVID-19 RT-PCR tests and implemented widely by most laboratories in many countries. These methods take advantages since they reduce resources, time, and overall costs required for a large number of samples. However, these methods could have more false negative cases and lower sensitivity. In order to maintain both accuracy and efficiency for different prevalence, we provide a novel pooling strategy based on the grid method with an extra pool set and an optimized rule inspired by the idea of error-correcting codes. The mathematical analysis shows that (i) the proposed method has the best sensitivity among all the methods we compared, if the false negative rate (FNR) of an individual test is in the range [1%, 20%] and the FNR of a pool test is closed to that of an individual test, and (ii) the proposed method is efficient when the prevalence is below 10%. Numerical simulations are also performed to confirm the theoretical derivations. In summary, the proposed method is shown to be felicitous under the above conditions in the epidemic.

## 1. Introduction

Group testing is a frequently used tool to identify an unknown set of defective (positive) elements out of a large collection of elements by testing subsets (pools) for the presence of defectives. The concept of group testing originated from the application of screening blood samples for syphilis during World War II, first suggested by Dorfman [1]. In Dorfman's method, samples are mixed together and tested in a single pool, and then, subsequent individual tests are made only if a pool is positive. Group testing strategy has been applied in other infectious diseases, including Chlamydia trachomatis, HIV, hepatitis B, malaria, and avian pneumovirus [2–9]. Recently, the idea of group testing (or sometimes pooling) has been validated for COVID-19 RT-PCR tests, implemented by labs in Israel [10, 11], German [12], and the United States [13, 14] and further studied in [15–23].

### 1.1. Related Works

So far, there have been two kinds of pooling strategies proposed for the diagnosis of SARS-CoV-2 with authorized RT-PCR tests. One is the Dorfman's method [19, 21, 22] (or called single pooling), where samples in the pools are pairwise disjoint and every patient belongs to exactly and only one pool; the other is multipooling where every patient can belong to more than one pool.

In the Dorfman's approach, if a pool test is negative, then all samples can be presumed negative with the single test, while if the test result is positive, then all the samples in the pool need to be retested individually. The advantages of this two-stage pooling strategy include preserving testing reagents and resources, reducing the amount of time required to test large numbers of samples, and lowering the overall cost of testing. Narayanan et al. [22] demonstrated the effectiveness of the Dorfman's method to accelerate testing for COVID-19. Hanel and Thurner [19] estimated the optimal pool size and the expected upper bound of missed infections, all as a function of the infection levels and the false negative/positive rates of PCR tests. Most laboratories turning to pool testing for more efficient COVID-19 surveillance use this approach.

Researchers found that pooling samples in certain ways, e.g., double pooling [17], bloom-filter pooling [15, 24], and the grid method [25], can help lowering the overall cost of testing. These studies reported that multipooling is significantly more efficient than the standard individual testing approach (reducing the total number of tests up to fourfold at 2% prevalence and eightfold at 0.5% prevalence [25]) and the single pooling approach in certain ranges of infection levels (30% improvement at 1.1% prevalence and at least 10% improvement all the way up to 5.4% prevalence [17]). The essence of the idea behind previous multipooling approaches is as follows: every patient belongs to two pools so as to be tested twice. For every patient, if both the pools test positive, then test the patient individually. Otherwise, that patient is considered to be clear.

Although they all share the same idea, there is a difference in the way of how they are designed. Designs based on the bloom-filter pooling [15, 24] rely on a random hash function and require a relatively complicated decoding, which could be one of the reasons why the use of such strategies is not popular. The grid method [25] is a two-dimensional pooling structure which can be represented as a matrix with fixed sizes, while the double pooling approach [17] divides the population into pools randomly. Among these strategies, the grid method is a simple pooling extension to existing SARS-CoV-2 testing protocols to boost efficiency and better utilize scarce resources.

### 1.2. The Grid Method

In [25], all samples of the library to be screened are arranged in a 2-dimensional grid of fixed sizes: a 96-well (8 × 12) plate and a 384-well (16 × 24) plate. One can then pool them according to the rows and the columns of the grid. Precisely, each row and each column give a pool, and then, we perform a test on each pool. Notice that two copies of the library are required at this stage. Then, in the second stage, all samples for which both the row and column which were tested positive are tested individually again to determine which individuals are positive. See Figure 1 for an example.

The double pooling approach such as the grid method not only improves the efficiency but also has another advantage that infected samples can be determined in an early stage. Under the described grid method, an infected sample will render its row and its column positive, so all the positive samples will be located immediately at the intersection of a positive row and a positive column. However, the reverse is not true. As shown in Figure 1, there can be many normal samples appearing in an intersection of a positive row and a positive column. In fact, if *x* samples are positive, then there are at most *x* rows and *x* columns tested positive (not exactly since two positive samples can be in the same pool), and *x*^2^ intersections are potentially positive. It is impossible to determine in the first stage which individuals are the exact *x* infected samples. To distinguish this, an additional test which is performed individually is necessary in the second stage.

However, there are obvious drawbacks to this approach which relies very much on the infection rate and sensitivity, although it has been proved more efficient than the classic Dorfman's method in a certain range of infection levels. The infection rate of the population can directly affect the number of tests performed in the second stage, which relies on the number of potential candidates leave behind the first stage. It is undesired if the number of such potential candidates is too many. However, this is an inevitable consequence of inflexible pool sizes in the grid method in [25].

Pooling samples reduce test sensitivity (to greater extents with larger pool sizes). In a study of testing the ability of the standard PCR test for detecting a single positive sample within a pool of negative samples, positive samples can still be well observed in pools of up to 32 samples and possibly even 64 with additional PCR cycles, with an estimated false negative rate of 10% [11]. Reported false negative rates of individual testings have ranged from less than 5 to 40 percent, although these estimates are limited, in part because there is no perfect reference standard for comparison [26–28]. False positive results are rare but have been reported with certain platforms [29] whereas false negative results can occur for numerous reasons, including suboptimal specimen collection, testing too early in the disease process, low analytic sensitivity, inappropriate specimen type, low viral load, or variability in viral shedding. Once a false negative outcome occurs in the process of the grid method, excluding those samples appearing in a negative test may lead to severe damage. The major concern for false negatives is someone who tests negative in a pool, thinking they are not infected, could unknowingly spread the virus into the community.

Another important feature is that a positive RT-PCR test for SARS-CoV-2 has more weight than a negative test because of the test's extremely high *specificity* 100% [30] but relatively moderate *sensitivity*. Specificity is the proportion of patients without disease who have a negative test, while sensitivity measures the proportion of actual infected samples that are correctly identified. Sensitivity and specificity can be confusing terms that may lead to misunderstanding.  Figure 2 explains these notions of statistical measures of test accuracy, including *false positive rate* (FPR) and *false negative rate* (FNR). Although (sensitivity, FNR) and (specificity, FPR) are simply the inverse of each other, to distinguish the notions on tests or strategies that we are talking about, sensitivity and specificity are used primarily for strategy outcomes while FNR and FPR are used for test outcomes.

### 1.3. Abbreviations

FNR:False negative rate (of an individual test or of a pool test),

FPR:False positive rate (of an individual test or of a pool test),

TFNR:True false negative rate = 1 − sensitivity,

TFPR:True false positive rate = 1 − specificity.

Previously mentioned, single pooling and multipooling approaches do not fully reveal potential advantages in terms of sensitivity. The reason is that, in a multipooling strategy, every sample (including infected ones) could be tested in more than two pools, and consequently, the probability of an infected sample being detected is increasing with respect to the number of pools it appears. Nevertheless, there is a relative lack of research to designs and analysis of pooling strategies going along with the benefit of improving sensitivity, which may lead to severe damage from the practical point of view. An interesting and important question is that “how to design a better pooling strategy with accurate case detection and efficient performance than individual testings?”. It is possible that performing several simultaneous or repeated tests could overcome an individual test's limited sensitivity; however, such strategies need validation [31]. In addition, it would raise efficiency concerns about performing tests several times.

The current study is aimed at proposing an easy-to-implement pooling strategy with both accurate case detection and efficient performance than the individual testing approach. Our approach, the triple grid method, is based on the two-dimensional grid method, but a big difference is that every patient is tested in three pools in the first round so as to offer more error-correcting capability. On the basis of data from more than 50 countries, we simulate and compare results among the standard individual-testing approach, the grid method, and the proposed triple grid method under a wide range of infection levels. Mathematical analysis points to the triple grid method being the best strategy in sensitivity if FNR of pool tests is not much worse than FNR of individual tests when FNR of individual tests is in the range [1%, 20%]. Moreover, taking into account the infection rate and error rates of the currently used PCR tests, we suggest a flexible pool size depending on the infection level to optimize the error-correcting capability, estimate the expected upper bound of missed cases in the strategy, and evaluate the benefits across both simulated and real data. An interactive web visualization of simulations is available at https://www.andylee.tw/covid19/.

## 2. The Triple Grid Method

### 2.1. Principle Aspect

Inspired by the grid method in [25], our triple grid method is aimed at reducing the chances of assessment errors caused by double pooling designs. Since the true positives are supposed to present as positive with high accuracy, the probability of frequent errors is relatively low. To discriminate between true and false positives, one or several more pools are needed. The following is the procedure of the triple grid method.

1. Four swabs are taken for each person. This is feasible since it was examined that up to 10 tubes are allowed [12]
2. Four *w* × *w* plates are prepared (the value *w* depends on the infection rate and will be discussed later), and each well, corresponding to a patient, in each plate contains a single sample obtained from a patient's swab. Formally speaking, a plate can be treated as a matrix [*m*_*ij*_] of size *w* × *w*
3. Test mixtures of all the samples in each row of the first plate, in each column of the second plate, and in each parallel diagonal of the third plate. That is, there are *w* row pools {*m*_*i*1_, *m*_*i*2_, ⋯, *m*_*iw*_} for 1 ≤ *i* ≤ *w*, *w* column pools {*m*_1*j*_, *m*_2*j*_, ⋯, *m*_*wj*_} for 1 ≤ *j* ≤ *w*, and *w* diagonal pools {*m*_1,*j*_, *m*_2,*j*+1_, ⋯, *m*_*w*−*j*+1,*w*_, *m*_*w*−*j*+2,1_, ⋯, *m*_*w*,*j*−1_} for 1 ≤ *j* ≤ *w*. Notice that the index is cyclic, and thus, the index *j* − 1 = 0 is equivalent to *j* − 1 = *w*.  Figure 3 demonstrates an example of *w* = 7
4. Every patient presents in at most one positive pool can be excluded; otherwise, individual tests are made for those with a relatively high risk (e.g., presenting in at least two positive pools or in three positive pools under certain scenario)

### 2.2. Practical Aspect

The first concern of applying this strategy is to choose the pool size *w*. By applying this approach, there are total 3*w* tests instead of *w*^2^ in the first stage, a significant reduction when *w* is large. However, this choice of *w* depends not only on the number of samples to be screened and technical limitations but also on the redundancy (the number of potential candidates to be confirmed in the second stage): if the number of infected samples is large, then there can be several samples which are clear but presenting in two or even three pools that contain an infected sample.

In this case, thinking simply all of the samples appearing in three positive pools are positive makes no sense and can cause several false positives. To distinguish them, more tests should be taken in the second round. Picking individual samples to retest in the second round is prone to not only efficiency but also reliability. It could lead to more unnecessary worries if staff wrongly declared a person who turned out not infected to be suspected and needed to confirm in the second round.

With this in mind, here we suggest choosing a number *N* of samples at most 1/*p* to test in a grid and set the pooling size $w=\left\lceil \sqrt{N}\;\right\rceil$, where *p* is the infection rate. A good reason of setting *N* ≤ 1/*p* is to limit the number of infected samples in the grids so as to reduce the number of tests required to do in the second round. If there is only one infected sample in the grid, then other samples appear in at least two negative pools unless some false positive test occurs. Therefore, all other samples can be declared to be virus-free with confidence since the false positive rate is very low in practice [30, 32]. As a consequence, no retests are needed if there is at most one infected sample in the grid, which is the most usual case by setting *N* ≤ 1/*p*. In fact, the triple grid strategy offers an error-correcting capability of one experimental error if there is only one infected sample in the grid. That means even if one error occurs (no matter false positive or false negative cases), the Diagnostic Algorithm below can successfully identify the only infected sample.

Note that throughout the above discussion there is a presumption that both *N* ≤ 1/*p* and $w=\left\lceil \sqrt{N}\;\right\rceil$. Based on the practical constraints of pool size in [11], which examined how diluting many negative samples with a confirmed positive sample would affect the test sensitivity of a single pool and suggested that 32 people (up to 64 people with more cycles) could be tested in a single pool with high sensitivity about 90% (that is, FNR 10%), we require the pool size *w* in an applicable range *w* ≤ 32; meanwhile, we also require *w* ≥ 4 because of efficiency concerns. That is,

(1) $$\begin{array}{c} w=\left\{\begin{array}{c} 4,\text{if }\left\lceil \sqrt{1/p\;}\;\right\rceil \leq 4,\\ 32,\text{if }\left\lceil \sqrt{1/p}\;\right\rceil \geq 32,\\ \left\lceil \sqrt{1/p}\;\right\rceil ,\text{otherwise}. \end{array}\right. \end{array}$$

The second concern is the criteria of how to select candidates who are suspected with a relatively high risk and need to retest in the second round. In our approach, each individual sample is tested thrice. Let *t*(*A*) denotes the number of positive pools a sample *A* appears and *N*_*j*_is the number of samples appearing in *j* positive pools, e.g., *N*_3_ = |{*A* : *t*(*A*) = 3}|. We suggest the following Diagnostic Algorithm:

(R1) When *t*(*A*) = 3, identify sample *A* as positive if *N*_3_ ≤ 3; otherwise, retest *A* individually and interpret the infection result based on the test.

(R2) When *t*(*A*) = 2, identify sample *A* as positive if *N*_3_ = 0 and *N*_2_ = 1; otherwise, retest *A* individually and interpret the infection result based on the test.

(R3) When *t*(*A*) ≤ 1, identify sample *A* as negative.

In general, a sample should be identified as positive firmly if it appears in three positive tests. But, in R1, we suggest retesting these samples when *N*_3_ is large to reduce false positive cases. The reason is that when *N*_3_ is large there are several infected samples in the grid, and in this case, it is likely that a number of normal samples are falsely claimed as positive only because they just appear in the intersections of positive pools.

Intuitively, testing a sample repeatedly helps in increasing the accuracy. But we find it is not the case to retest a sample *A* with *t*(*A*) = 2 in R2 when *N*_3_ = 0 and *N*_2_ = 1. The crucial idea is that doing imperfect tests on an infected sample could possibly yield negative results. In this case, it is more likely that the sample *A* is an infected sample with one false negative result. By limiting the average number of infected samples in the grids, cases with one infected sample and one false negative outcome (like the mentioned sample *A*) would be one of the most frequent cases with error outcomes. But that error can be detected and corrected by our algorithm. This is the main reason of why the proposed method significantly improves the overall sensitivity, as compared with the two-dimensional grid method. More details will be explained later in Mathematical Analysis.

Remark that *t*(*A*) = 2 is a natural threshold to determine whether a sample A is infected with a relatively high probability. If it is one, then an underfitting situation occurs frequently since every sample appearing in a pool with a positive sample satisfies these criteria. In the case of only one infected sample in the grid, this implies a number 3(*w* − 1) of suspected candidates even if no false negative occurs. If it is three, then an overfitting situation occurs since every true positive sample cannot pass the standard in the first round. An approach to retesting these samples all the time is low efficiency.

## 3. Simulation Results

It may be useful to give an example to illustrate these theoretical considerations: we could envisage using the pooling approach to screen the libraries with various population wide infection levels, for example, of *p* = 1% at present 10,000,000 samples. According to the triple gird procedure, we set *N* = 1/*p* = 100, implying that a total of 100,000 simulations were executed with pool size $w=\left\lceil \sqrt{N}\;\right\rceil =10$. Suppose FNR of a single test/pool is 5%/10% and FPR of a single test/pool is 0.1%/0.1%. A simulation result returns the usage ratio 35.92% (3,591,952/10,000,000) with sensitivity 95.73% (94,318/98,518) and specificity 99.99% (9,900,557/9,901,482) for the Diagnostic Algorithm of the triple grid approach. That points to relatively lower true false negative rate (TFNR) 4.27% and true false positive rate (TFPR) 0.01% of the procedure than FNR 10% and FPR 0.1% of a pool, respectively.

Under the same conditions of FNR and FPR as the previous case study, if the infection rate increases to *p* = 4% and thus *w* = 5, then a simulation result returns the increase of the usage ratio 65.70% (1,642,474/2,500,000) with comparable sensitivity 96.03% (96,658/100,655) and specificity 99.95% (2,398,150/2,399,345). The pool size *w* = 5 remains all the way up to infection levels 6.24%, and in this case, the usage ratio increases to 72.37% with sensitivity 95.37% and specificity 99.88%. For an infection level of 10% with the pool size 4, the usage ratio increases to 92.05% with a slightly better sensitivity 95.29%; for higher infection levels with the same pool size 4, the triple grid method is of little use in practice because additional numerous technical barriers are removed but only to obtain almost no cost reduction.

The simulations were done by using a sampling approach: drawing samples from a Bernoulli distribution with a probability equal to the assumed infection rate *p*. All draws were independent, and a total of 100,000 runs were executed to smooth over any sampling noise. The results of our triple grid approach are compared with the individual testing approach and the previous grid approach, and a simpler interactive version of simulations with adjustable parameters such as infection levels, pool sizes, and error rates can be experienced in our web interface https://www.andylee.tw/covid19/.

Figure 4 compares the efficiency gain by applying our procedure with those obtained separately from the individual-testing procedure and the grid method. As the grid size is selected inversely proportional to the square root of the infection rates, it is an expected decrease of the efficiency gain with an increasing infection rate.

We also used the simulations to evaluate the expected number of missed cases in our strategy and evaluate the benefits across both simulated and real data. We found that both the grid method [25] and the triple grid method improve the efficiency of the number of tests when the infection level is less than 26.77% (Qatar) and 11.74% (Kuwait), respectively. However, the grid method results in an expected 1,511,345 missed cases, which is significantly more than 329,588 missed cases of the individual testing method over all data of the 52 countries. When the infection level is less than 0.43% (Lithuania), the strategy which performed best on both efficiency and sensitivity across countries is the triple grid method; when the infection level is less than 11.74% (Kuwait), it is the triple grid method that performed best on sensitivity. These findings suggest that the triple grid approach is a straightforward compromise between sensitivity and efficiency if the infection level is low (less than 11.74%). Using testing and positive test estimates from Our World in Data [32], we chose an accuracy-optimal testing strategy per country from between individual testing method, the grid method, and our triple grid method, where an accuracy-optimal strategy means that the one minimized the number of missed cases. This resulted in an expected total of 75,193,229 tests (1.4x improvement) and an expected total of 287,708 missed cases (1.14x improvement) to retest everyone who has previously been screened for SARS-CoV-2 (see Figure 5).

## 4. Mathematical Analysis

In this section, we provide estimations for the number of samples to retest in the second round and the FNR of our procedure, and a proof of why the triple grid method would be able to successfully identify the only one infected sample even in the case of some errors happened.

### 4.1. Notations

*p*:The population infection rate,

*N* = 1/*p*:The number of samples in a grid,

$w=\sqrt{1/p}$ :The pool size,

*γ*_0_:FNR of individual tests,

*γ*_1_:FNR of pool tests,

*X*:A random variable of the number of infected samples in a grid.

For ease of analysis, throughout the rest of this section, we assume false positive rate FPR = 0% for both individual tests and pool tests and ignore the constraint that *N* and *w* are integers. All the following analysis is based on the assumption that the random variable *X* has a Poisson distribution. A discrete random variable *X* is said to have a Poisson distribution with parameter *λ* > 0, if it has a probability mass function given by

(2) $$\begin{array}{c} \mathrm{Pr}\left(X=k\right)=\frac{\lambda^{k}e^{-\lambda }}{k!}, \end{array}$$

where *k* is the number of occurrences and *λ* is equal to the expected value of *X* and also to its variance.

### 4.2. Computation of the Expected Number of Samples to Retest in the Second Round

The theoretical analysis gives consistent results with simulations on the efficiency of our procedure. Due to a particular choice of $w=\sqrt{1/p}$ on the triple grid method, infected samples occur once in every grid on average. To calculate the probability of the event that *X* = 0, 1, 2, ⋯, infected samples occur in the grid, assuming the Poisson model is appropriate. Actually, the Poisson distribution with parameter *λ* = *Np* is an approximation of the binomial distribution and applies well in the capacity *p* ≤ 0.05 and *N* ≥ 20 [33], which is in our case *w* ≥ 5.

Because the expected rate of occurrences is one infected sample per grid, we have *λ* = *Np* = 1, and thus, the probability Pr(*X* = *k*) = *λ*^*k*^*e*^−*λ*^/*k*! = 1^*k*^*e*^−1^/*k*!. By simple calculation, the following estimations are obtained:

(3) $$\begin{array}{c} \mathrm{Pr}\left(X=0\right)=\frac{1^{0}e^{-1}}{0!}=\frac{e^{-1}}{1}\approx 0.368,\\ \mathrm{Pr}\left(X=1\right)=\frac{1^{1}e^{-1}}{1!}=\frac{e^{-1}}{1}\approx 0.368,\\ \mathrm{Pr}\left(X=2\right)=\frac{1^{2}e^{-1}}{2!}=\frac{e^{-1}}{2}\approx 0.184,\\ \mathrm{Pr}\left(X=3\right)=\frac{1^{3}e^{-1}}{3!}=\frac{e^{-1}}{6}\approx 0.061,\\ \mathrm{Pr}\left(X=4\right)=\frac{1^{4}e^{-1}}{4!}=\frac{e^{-1}}{24}\approx 0.015. \end{array}$$

Accordingly, most cases (about 73.6%) occur with at most one infected sample in the grid, and in this case, all samples can be successfully classified even if one error occurs (see discussion below for error-correcting capability). There are some cases (18.4%) having two infected samples, which additionally lead to at most 6 normal samples locating at intersections of two out of the six positive pools if error-free. This case contributes to at most 1.2 (expected number) samples needed to retest. As the probability of the rest cases is low, it affects not much (at most an estimated number of 3 samples to retest) even taking into account *γ*_1_ in the level of 10%. We found that pooling in this way leads to only a constant 5 increase in the total number of samples to retest in the second round. Remark that the simulation results obtained a number less than 3 on average.

### 4.3. Error-Correcting Capability

In the previous grid method [25], an infected sample renders both its row and column positive, so all the positive samples will be located immediately at the intersection of a positive row and a positive column. If there are more than one infected sample, then simply identifying samples located at the intersection of a positive row and a positive column as positive will cause several false positives. Retests are necessary to distinguish them. On the other hand, if there is at most one infected sample in the grid, then two pools are positive (one in rows and the other in columns), and we can identify the intersecting sample as positive firmly. Unfortunately, if one error occurred in one of the corresponding row and column, which means only one positive pool in the grid, then it is impossible to determine which sample is positive without any further information. To improve the efficiency of experiments, several methods of screening have been studied from the point of view of mathematics [34–36].

Recall that in R2 of the Diagnostic Algorithm, we suggest not retesting the only sample *A* with *t*(*A*) = 2 when *N*_3_ = 0. The reason is that the proposed triple grid design can identify the only one infected sample even if one error occurs. Observe that every sample appears exactly at the intersection of three pools (between columns, rows, and parallel diagonals), which can be interpreted geometrically as every point lies on the intersection of three lines. When one error occurs, there are still two positive pools, and we can use the two lines to locate which sample is positive. By simple calculation, one can find that at most one false negative error occurs in the three supposed-to-be positive pools with high probability unless *γ*_1_ is extremely high.

From the simulation results in Figure 5, we found that the one error correcting property plays an important role in improving the rate of the number of missed cases (improvement from 4% to 12% if the infection rate is low).

### 4.4. Computation of True False Negative Rate

To estimate the number of missed cases, we derive the probability that an infected sample is misclassified as negative by the Diagnostic Algorithm of the triple grid approach, that is, true false negative rate (TFNR). According to the Diagnostic Algorithm, there are four potential cases, and it suffices to consider three cases from the above discussion:

1. Those *A*'s with *t*(*A*) ≤ 1

The probability of at least two false negative errors out of three supposed-to-be positive pools is *γ*_1_^3^ + 3*γ*_1_^2^(1 − *γ*_1_) = *γ*_1_^2^(3 − 2*γ*_1_).

(2) Those *A*'s satisfying *t*(*A*) = 2, *N*_2_ + *N*_3_ ≥ 2, and negative retest outcome

The probability of one false negative error out of three supposed-to-be positive pools is at most 3*γ*_1_(1 − *γ*_1_)^2^, ignoring the condition of *N*_2_ + *N*_3_ ≥ 2. The probability of retesting such a sample *A* and remaining negative would be 3*γ*_1_(1 − *γ*_1_)^2^*γ*_0_.

(3) Those *A*'s satisfying *t*(*A*) = 3, *N*_3_ ≥ 4, and negative retest outcome

The assumption of FPR = 0%, *N*_3_ ≥ 4 implies at least four infected samples appearing in the grid, which has probability Pr(*X* ≥ 4) ≤ 2%. Thus, the probability of retesting such a sample *A* and remaining negative is at most 0.02*γ*_0_. This value is relatively small as compared with the previous two in the range of 2% ≤ *γ*_0_ ≤ 10%.

The expected true false negative rate of our procedure can be computed according to the above discussion. For example, when *γ*_0_ = 5% and *γ*_1_ = 10%, the probability that at most one false negative occurs among three positive pools is 72.9% + 24.3% = 97.2%, and the probability of at least two false negative errors out of three positive pools is reduced down to 2.7% + 0.1% = 2.8%, which is the first case. As for the other two cases, it is around 1.2% + 0.1% = 1.3%; thus, we have the expected TFNR 4.1% of our approach, a number less than FNR of Dorfman's method (10%) and FNR of individual testing approach (5%). In certain ranges of *γ*_0_ and *γ*_1_, we find that applying our triple grid method significantly improves TFNR (see Figure 6).

## 5. Discussions

We propose an alternative group testing scheme with an error-correcting capability to improve sensitivity while maintaining the benefit of reducing cost. These are not meant to be a replacement for individual testing and other pooling approaches. There are numerous practical concerns that must be considered. Accuracy of RT-PCR tests in clinical practice varies depending on the quality of sampling, stage of disease, and degree of viral multiplication or clearance [37]. There may be many medical, testing, or supply chain reasons such pooling strategies will not work, including mixing samples from multiple individuals in a single tube risks contamination and picking individual samples to retest is prone to pipetting errors (see [25] for more details). All of these practical concerns that should be considered in any existing pooling strategy must be considered thoroughly when applying our triple grid method.

It is known that one should never pool samples above a prevalence of above 30%; however, in the triple grid method, the threshold is below 10%, a comparable result with that suggested in the grid method. The efficiency gain increases when the prevalence decreases from 10% all the way down to 0.1%. This means that the proposed method and the existing double pooling approaches have similar implementation scenarios and could only be used with pooled samples from low-risk individuals without known or suspected COVID-19.

The availability of accurate laboratory tools for COVID-19 is essential for case identification, contact tracing, and optimization of infection control measures. False negative results can occur for numerous reasons [26, 38]; however, there are several possible scenarios that pooling a sample in several tests such as our strategy would not work well to avoid such false negative results, including suboptimal specimen collection, testing too early in the disease process, and low viral load. Risks to a patient of a false negative result include delayed or lack of supportive treatment and lack of monitoring of infected individuals and their close contacts for symptoms resulting in an increased risk of spread of COVID-19 within the community. This kind of information matters when people take a test because how this uncertainty about the tests is communicated influences how people understand their test results, which in turn has the potential to influence their decisions and actions.

A feature of the proposed triple grid method is that the pool size *w* is flexible and relies on the prior knowledge of the prevalence *p*, which is a major reason for improving the sensitivity when applying our method. However, this raises clinical barriers to choosing the pool size because in reality it is usually difficult to have the information of an accurate infection rate of a population, and the infection rate usually varies with time and with space. That, in turn, suggests that paying attention to the need for good estimation of the infection rate of a population to be tested will be important in managing diagnostic tests.

We assume that samples are distributed at random and independently. However, sample collection for this approach might be conducted through contact tracing and door-to-door sampling, where we expect cohabitation. In these cases, the assumption of lack of correlation of test status between individuals does not hold.

This study is limited in that it was only analyzed mathematically but not performed in any laboratory. Additional experimental data are thus required to validate this approach in practice.

## 6. Concluding Remarks

To conclude, this paper provides an alternative group testing scheme with an error-correcting capability to improve sensitivity while maintaining the cost reduction benefit of the existing pooling strategies. However, besides the mentioned practical concerns, whether or not to use this triple grid method depends on the requirement of the efficiency and also the tolerance of the number of missed cases. Let us consider the simplest case that testing a pooled sample does not change the false positive and false negative rates of the test and assume FPR = 0%. For the case of the infection level 1% and FNR 5%, the usage ratios are about 20%, 22%, and 32%, and the sensitivities are about 90%, 86%, and 98% for the Dorfman's method (pool size 10), the grid method (96-well plates), and our method (pool size 10), respectively. For an infection level of 5% with the same condition FNR 5%, the usage ratios are about 45%, 36%, and 68%, and the sensitivities are about 90%, 85%, and 98% for the Dorfman's method (pool size 5), the grid method (96-well plates), and our method (pool size 5), respectively. For the same FNR and an infection level of 10%, the usage ratios increase to 65%, 59%, and 94% with comparable sensitivities 90%, 86%, and 97%.

That in turn suggests that the proposed triple grid method being a straightforward compromise between efficiency and sensitivity can offer a high-quality diagnosis to reduce the number of missed cases when the infection level is low, and pooling sample does not affect FNR of the tests. If pooling samples increase FNR of the tests, then our strategy provides expanded benefits for maintaining sensitivity. For example, for an infection level of 5% with FNR of individual tests = 5% and FNR of pooled tests = 10%, the usage ratios are about 45%, 35%, and 69%, and the sensitivities are about 85.5%, 76.6%, and 95.6% for the Dorfman's method (pool size 5), the grid method (96-well plates), and our method (pool size 5), respectively.

High-sensitivity pooling strategies such as those proposed here will be valuable in expanding testing capacity and precisely locating potentially infected individuals. In some countries like U.S., emergency use authorizations (EUAs) have been issued to authorize the tests for use with pooled anterior nasal specimens for screening when used as part of a serial testing program. Tests authorized for use can only be used in such laboratories that meet certain requirements, e.g., sensitivity 95% [39], to perform high complexity tests to detect SARS-CoV-2. While there are numerous medical, testing, or supply chain barriers left to overcome, we anticipate that this proposed method offers an alternative option for any laboratory that wishes to use pooling samples for adequate testing capacity but fails to meet the high-sensitivity requirement.

Although we assumed FPR is 0%, as suggested in [30], and did not address this issue throughout the mathematical analysis, we found that the triple grid method improves not only the sensitivity but also the specificity in some cases. These findings were obtained by simulation results and can be examined by adjusting the value of FPR via our web interface https://www.andylee.tw/covid19/. We encourage further work into rigour statistical tests to evaluate this more thoroughly.

We see a great potential of applying such a pooling strategy for rapid scaling up COVID-19 testing. Reopening is an urgent and huge challenge to most countries in the world and is a likely scenario to apply our pooling strategy. According to [31], diagnostic testing will help in safely opening the countries, but only if the tests are highly sensitive; moreover, it will also be important to develop methods for estimating the pretest probability of infection for asymptomatic and symptomatic people. In fact, our approach achieves nice sensitivity even higher than the individual testing approach in certain ranges of conditions. With better estimations of the pretest probability of infection for travellers from different areas, among individuals with a low probability of infection, this methodology might be particularly well-suited to traveller screening through reliable RT-PCR tests for COVID-19.

## Figures and Tables

**Figure 1:** Given a population of 96 patients, infected samples are marked bold, and there are five infected samples in the 96-well plate. A single pooling approach of pool size 8 can be represented by 12 pools, each in a column, as demonstrated in (a), while the grid method tests not only the 12 vertically parallel pools but also 8 horizontally parallel pools as shown in (b). In the single pooling, there are five positive pools if all tests are error-free, and thus in the second, all the 40 samples appearing in these five pools need to retest individually, which yields a total of 52 tests across the 96 individuals and a 44/96 ≈ 45.8% improvement over the standard individual testing. However, in the grid method, only those samples appearing in both positive outcomes will be tested individually again to assess what status of COVID-19 it may have, so those appearing in a negative row or column can be excluded. Only those samples with bold circles will go to the second round. Therefore, there are total 40 tests across the 96 individuals being tested (8 rows plus 12 columns plus 20 remaining individuals), a 56/96 ≈ 58.3% (12/52 ≈ 23.0%) improvement over the standard individual testing (the single pooling), respectively. Note that the discussion above is made under the assumption that the experimental scenario is error-free, which is obviously not the case in the real world. Things become much more complicated if some test errors occur in the first stage of the grid method.

**Figure 2:** The notion of sensitivity/specificity and TFNR/TFPR.

**Figure 3:** On three 7 × 7-well plates, pools of samples from each row, each column, and each parallel-shifted diagonal are tested in the first round. Totally, 7 + 7 + 7 = 21 pools are tested in this case. Every individual will be tested in three different pools associated with three corresponding swabs. As false negative rate of a single pool is low (about 10% examined in [11]), the probability of more than one false negative error out of the three pools is relatively lower. Thus, individuals for which at least two pools tested negative are not retested further in the second round.

**Figure 4:** Comparisons of the numbers of tests performed by our procedure, the grid method (96 wells), and the individual testing method. The efficiency of our procedure increases when applying in libraries with a low infection rate and can be better than that of the grid method as the infection rate is less than 0.5% (which means the pooling size is larger than 15).

**Figure 5:** Comparison of pooling strategies, individual testing method, the grid method (96-well), and the triple grid method, across countries. Across 52 countries with available data of cases and tests for COVID-19, the estimated numbers of tests and missed cases under a given condition that (FNR 5% and FPR 0.1% for individual tests, FNR 10% and FPR 0.1% for pool tests) are provided. Data of cases and tests for COVID-19 are collected from Our World in Data [32] (to the date 06/30/2020). The data in this table are sorted according to the value of the infection level in a nondecreasing ordering. Colored values are the best among the three considered methods.

**Figure 6:** Improvement percentage of expected false negative rate of our procedure to the individual testing method. For ease of analyzing the relation of FNR among the considered methods, the estimation is done by assuming FPR = 0 although it is a parameter adjustable in our model and the web interface. The *x*-axis indicates FNR of individual testing method, the *y*-axis represents FNR of the Dorfman's method, and the cell value is the estimated percentage of improvement of FNR of our procedure to individual testing method. For example, when FNR (individual test) is 0.05 and FNR (pool) is 0.1, it gains an estimated 20% improvement upon the false negative rate by using our strategy, i.e., TFNR ≈ 0.04.

## Data Availability

The cases and tests for COVID-19 data used to support the findings of this study are included within the article.
